# Crowd Control: Effects of Physical Crowding on Cargo Movement in Healthy and Diseased Neurons

**DOI:** 10.3389/fncel.2019.00470

**Published:** 2019-10-25

**Authors:** Vidur Sabharwal, Sandhya P. Koushika

**Affiliations:** Department of Biological Sciences, Tata Institute of Fundamental Research, Mumbai, India

**Keywords:** physical crowding, axonal transport, neuron, neurodegeneration, cytoskeleton, organelles, molecular motors

## Abstract

High concentration of cytoskeletal filaments, organelles, and proteins along with the space constraints due to the axon’s narrow geometry lead inevitably to intracellular physical crowding along the axon of a neuron. Local cargo movement is essential for maintaining steady cargo transport in the axon, and this may be impeded by physical crowding. Molecular motors that mediate active transport share movement mechanisms that allow them to bypass physical crowding present on microtubule tracks. Many neurodegenerative diseases, irrespective of how they are initiated, show increased physical crowding owing to the greater number of stalled organelles and structural changes associated with the cytoskeleton. Increased physical crowding may be a significant factor in slowing cargo transport to synapses, contributing to disease progression and culminating in the dying back of the neuronal process. This review explores the idea that physical crowding can impede cargo movement along the neuronal process. We examine the sources of physical crowding and strategies used by molecular motors that might enable cargo to circumvent physically crowded locations. Finally, we describe sub-cellular changes in neurodegenerative diseases that may alter physical crowding and discuss the implications of such changes on cargo movement.

## Introduction

Neurons are amongst the longest cells in most organisms, with lengths up to 1 m in humans (Fletcher and Theriot, 2004). This necessitates an efficient transport system that can move material from the cell body to distal processes. Some organelles, like endosomes, may have diameters up to 5 μm which are similar to the diameter of neuronal processes (200 nm to 20 μm) within which they move (Takamori et al., 2006; Misgeld et al., 2007; Assaf et al., 2008; Encalada and Goldstein, 2014). Thus, neurons may occasionally have local physically crowded regions where cargos that are similar in diameter to the neuronal process may stall.

Physical crowding is an outcome of a large number of macromolecules and organelles present in the cytosol of cells. A dense cytoskeletal network, pre-existing intracellular organelles, and a high concentration of proteins imply that the entire cellular volume in a given region is not always accessible to soluble molecules or organelles that move into a region. In line with previous literature, we refer to organelles, the cytoskeleton, and proteins as crowding agents. The volume not available is known as the excluded volume. The average concentration of proteins within a cell ranges from 17 to 35% by dry cell weight (Fulton, 1982). This concentration, along with an average size of about 50 kDa for typical soluble globular proteins, suggests that proteins are on an average closer to each other than their radius of gyration (Chang et al., 1987; Luby-Phelps, 1999). Macromolecular crowding describes the effect of proteins or complexes (e.g., microtubules, proteasomes) that exclude other small molecules from the space that they occupy. The presence of PEG of ∼2.5 nm or ∼20 nm radius leads to reduced association equilibria between TEM1-β-lactamase and β-lactamase inhibitor protein *in vitro* compared to solutions lacking PEG (Kozer et al., 2007; Zhou et al., 2008). This reduced association is thought to arise from the reduced rate of diffusion of the reactants (Kozer et al., 2007), perhaps due to reduced available solution space. The relative decrease in the diffusive movement for any diffusing molecule in the cytosol as compared to water arising both from macromolecular crowding and the viscosity of the cytosol is termed as microscopic viscosity (Lavalette et al., 1999). The microscopic viscosity is governed both by the concentration and the interactions between constituents of the solution (Lavalette et al., 1999). The microscopic viscosity of the cytosol will directly influence the diffusive properties of each molecule in the cell.

Crowding-related challenges are likely faced by all cells (Luby-Phelps, 1999), but are particularly relevant in neuronal processes with a narrow axonal diameter, the narrowest of which can be as low as 160 nm in diameter in vertebrates (Graf von Keyserlingk and Schramm, 1984; Perge et al., 2012; Fischer et al., 2018) and 100 nm in diameter in invertebrates (Chalfie and Thomson, 1979; Graham et al., 1986), both smaller than the known diameters of some organelles (Zhang et al., 1998; Encalada and Goldstein, 2014; Fischer et al., 2018). Additionally, neuronal processes have a high density of cytoskeletal elements (Osborn et al., 1978). Microtubules (MTs) and neurofilaments in neurons have been reported to have an average separation between them of about 25–100 nm (Osborn et al., 1978; Chalfie and Thomson, 1979). By contrast in non-neuronal cells, some MTs can be closely spaced but several are separated by >200 nm (Friede and Samorajski, 1970). Physical crowding is especially important when molecules, macromolecular complexes, and organelles need to move and position themselves within neuronal processes. Active transport that is dependent on molecular motors (Vale et al., 1985; Schroer et al., 1989; Mehta et al., 1999) is one strategy to circumvent crowding that leads to fast transport within a cell. However, active transport also faces physical challenges, such as availability of free tracks for transport (Shemesh et al., 2008) and crowded regions in the cytosol due to organellar exclusion (Mackey et al., 1981). Models of some neurodegenerative diseases are associated with decreased organelle velocity, organellar displacement, and increased organelle stalls (Gunawardena and Goldstein, 2001; Stamer et al., 2002; Pigino et al., 2003; Roy et al., 2005; Kang et al., 2014; Kreiter et al., 2018). Increased physical crowding by proteins, cytoskeletal polymers, and stalled membranous organelles in neurodegenerative diseases can all contribute to reducing cargo movement, thereby exacerbating the progression of neurodegenerative phenotypes.

Although there are many different sources of crowding in a neuron, how each source affects the movement of other classes of moving proteins, polymers, or organelles is currently unclear. This review examines existing evidence that suggests that physical crowding may influence cargo movement and the potential strategies that allow cargo to move despite crowding effects. The review concludes with possible experiments that may help delineate the role of physical crowding in influencing cargo movement in neurons.

## Physical Barriers to Diffusive and Active Cargo Movement

The location where some proteins or organelles function can be distant from the cell body in neurons (DeLorenzo and Freedman, 1978). Consequently, their transport through either diffusive or active (ATP dependent) mechanisms is essential. The different sources of physical crowding include: microscopic viscosity, macromolecules, organelles, diameter of the neuronal process, and cytoskeletal polymers. Some of these crowding agents may preferentially affect active over diffusive movement and are discussed below.

### Crowding Effects on Diffusion

The local environment can influence the diffusion of molecules via (i) reduction in apparent diffusion coefficients due to increased microscopic viscosity of the cytosol (Figure 1C) (Luby-Phelps, 1999; Zhou et al., 2008) and (ii) excluded volume effects arising from the presence of macromolecules and polymers such as actin, neurofilaments, and MTs (Figures 1, 2) (Luby-Phelps, 1999). Soluble proteins can diffuse at rates ranging from 0.02 to 50 μm^2^/s (Luby-Phelps, 1999). Increasing the viscosity of an aqueous solution by adding a large molecular weight polysaccharide, Ficoll 70, leads to reduced diffusion coefficients for several types of molecules (Dix and Verkman, 2008). A similar 4–100 times reduction in diffusion coefficients of proteins compared to their diffusion coefficients in water is observed in the cytosol (Luby-Phelps, 1999; Verkman, 2002). A decreased diffusion coefficient not only affects the movement of molecules but may also reduce reaction rates of fast reactions owing to reduced rates of bimolecular association (Zhou et al., 2008).

**FIGURE 1:** Schematic representation of sources of physical crowding in the axon. Magnified view of features that contribute to crowding shown in insets. **(A)** Actin cortical rings, deep actin. **(B)** Neurofilaments can physically crowd the neuron by excluding organelles and small molecules. **(C)** High concentration of soluble proteins and narrow axonal geometry can lead to a local increase in viscosity. **(D)** Stalled cargo can physically impede the movement of motile cargo and diffusive proteins. **(E)** The MT bundle can exclude organelles but may allow diffusion of small proteins.

**FIGURE 2:** Electron micrograph of myelinated axons from Central Nervous System (CNS) and Peripheral Nervous System (PNS). **(Top panel)** Some myelinated axons in the CNS have mitochondria (M) that can be up to half the diameter of the neuronal process. In the magnified view on the top right, we can see a number of microtubules (solid arrows) and neurofilaments (arrowheads). **(Bottom panel)** Small caliber axons in the Remak bundles (R) can be as thin as 200 nm. We also see the axon filled with mitochondria (M), microtubules (solid arrows), neurofilaments (arrowheads) and vesicles. Reprinted with permission from *Frontiers in Neuroscience*, 12, (2018) p. 467 (Stassart et al., 2018).

Additionally, protein diffusion can be retarded by the cytoskeletal network, such as at the axon initial segment (AIS) of the neuron that has a high concentration of F-actin and β-spectrin (Li et al., 2005; Song et al., 2009; Jones et al., 2014). Dextrans of 70 kDa injected in the cell body are restricted to the somatodendritic region, as opposed to smaller 10 kDa dextrans that freely diffuse in the axon (Song et al., 2009). The exclusion of 70 kDa dextran depends on F-actin that can form a physically crowded barrier or sieve at the AIS. Although as yet unexplored, the bundle of microtubules present in axons may also reduce the available volume for free diffusion (Wortman et al., 2014). However, microtubule depolymerization by nocodazole has not demonstrated a change in diffusion coefficients of small molecules like water (Colvin et al., 2011) or GFP (Song et al., 2009). The solute size where microtubules may be able to act as a crowding agent is unclear.

### Crowding Effects on Active Transport: Microtubules

Active transport leads to fast movement of molecules over long distances (Nitta and Hess, 2005; Ribeiro and de Wit, 2017). This type of transport utilizes molecular motors that walk on either actin or MT tracks (Vale et al., 1985; Schroer et al., 1989; Mehta et al., 1999). MT motors play a major role in long-distance transport in neurons. There are three major sources of crowding experienced by cargo trafficked on MTs: (i) molecular crowding on tracks, (ii) crowding due to organelles in the vicinity of moving cargo, and (iii) drag from the axonal cortex.

Sources of crowding on MT tracks may include MT-associated proteins (MAPs), cargo stalled along the tracks, or protein/organelles at MT ends. Since the average length of MTs is shorter than that of axons, MTs are present as an overlapping staggered array within the neuronal process (Chalfie and Thomson, 1979; Bray and Bunge, 1981; Yogev et al., 2016). Thus there are numerous MT ends along the neuronal process, locations where both motors and cargo are shown to stall (Lipowsky et al., 2001; Leduc et al., 2012; Yogev et al., 2016). Additionally, neuronal processes in an organism are flexible to allow movement (Krieg et al., 2017; Datar et al., 2019). A dynamic reorganization of the MT bundle may lead to non-uniform cargo stalling that further leads to rapid changes in local physical crowding in the axon (Ahmed et al., 2012). To maintain cargo transport with dynamic overlapping MT tracks, a cargo must navigate multiple MTs to reach its destination, for instance, the synapse. Ability to move across tracks in part depends on the availability of a free track for motor attachment and movement.

Microtubule associated proteins, such as Tau and MAP2 (Lakadamyali, 2014), or tubulin post-translational modifications, like polyglutamylation or tyrosination (Sirajuddin et al., 2014; Lessard et al., 2019), are known to physically compete with or affect the affinity of MT motors for binding sites on the MTs respectively (Hagiwara et al., 1994; Stamer et al., 2002; Vershinin et al., 2007). However, the extent to which each MAP competes with MT motors can differ (Gumy et al., 2017). Since MAPs may be distributed differentially on the minus and plus end of a given MT (Qiang et al., 2018), movement of MT motors may vary depending on their location on the MT (Dixit et al., 2008; Monroy et al., 2019). As an example, the plus TIP complex that forms at the plus end of MTs may physically compete with MT motor binding, forcing the release of MT motors and associated cargo from the MT plus end (Akhmanova and Steinmetz, 2015). *In vitro*, kinesin motors are also known to physically crowd the plus end of MTs leading to a slowing of other kinesins approaching the plus end (Telley et al., 2009). Therefore, MT motors face many obstacles on the transport path to facilitate the active movement of cargo.

### Physical Crowding Effects on Active Transport: Organelles

Transported cargo that varies in size from 0.04 to 2 μm (Zhang et al., 1998; Encalada and Goldstein, 2014; Fischer et al., 2018) can also be physically obstructed by objects present in its vicinity. These include stationary cargo in close proximity, actin-rich regions along the axon (Sood et al., 2018), and trapping of cargo by the actin cytoskeleton in the dendrite (Bommel et al., 2019). A subset of different stationary cargo has been observed in the neuronal processes of a variety of neurons (Kang et al., 2008; Tang-Schomer et al., 2012; Iacobucci et al., 2014). These stationary cargos can themselves physically impede the transport of any moving cargo that encounter them, irrespective of the cargo type, thereby leading to a local build-up of stalled cargo (Sood et al., 2018). Moreover, increased cargo stalling and reduced cargo run length are observed in crowded regions that are enriched in actin (Sood et al., 2018; Bommel et al., 2019). Therefore, both actin-rich regions and stationary cargo at actin-rich regions may act as local crowding agents for moving membrane-bound organelles (MBOs) irrespective of cargo type.

### Physical Effects on Active Transport: The Axonal Cortex

Cargos may also face increased drag due to interaction with the axonal cortex. In neurons, the axonal diameter ranges from ∼160 to 20 μm in humans (Graf von Keyserlingk and Schramm, 1984; Perge et al., 2012), and ∼100 to 350 nm in *Caenorhabditis elegans* (Chalfie and Thomson, 1979; Graham et al., 1986). Cargos that are transported in axons may occasionally contact the axonal cortex (Topalidou et al., 2012; Narayanareddy et al., 2014; Wortman et al., 2014). For instance, in axons, retrogradely moving lysotracker-marked vesicles induce local stretching of the plasma membrane of the axon (Wang et al., 2018). This could lead to increased drag, and may cause moving organelles to encounter greater stiffness from the proximate axonal cortex compared to stiffness encountered within the cytosol. Consistent with this hypothesis, the speed of large organelles in neuronal processes is shown to reduce with increasing organelle size and reducing axonal diameter (Narayanareddy et al., 2014; Leite et al., 2016).

In conclusion, there are many crowding agents in the neuron that can impede the movement of molecules within the neuronal process (Pannese et al., 1984; Luby-Phelps, 1999; Sood et al., 2018; Vassilopoulos et al., 2019). Cytosolic diffusion is affected by the viscosity of the medium where the cytoskeletal filaments themselves can act as molecular sieves (Lewis et al., 2009; Song et al., 2009). On the other hand, active transport by molecular motors on MT tracks is affected by crowding on MT tracks (Hagiwara et al., 1994; Akhmanova and Steinmetz, 2015; Gumy et al., 2017), by the axonal plasma membrane (Narayanareddy et al., 2014; Leite et al., 2016; Wang et al., 2018), organelles, and cytoskeletal filaments near the tracks (Figures 1B,D,E) (Sood et al., 2018; Bommel et al., 2019). Both diffusion and motor-dependent movement face physical constraints that cargo must circumvent for steady transport.

## Strategies for Bypassing Crowding Depending on the Type of Neuronal Cargo

Neuronal cargos can vary in size and chemical composition. However, each type of cargo achieves long-range transport that can bypass physical crowding. Small molecules may be transported along neuronal processes by diffusion, active transport, or a combination of both. This may prove sufficient for small proteins, however, large protein complexes with potentially slower diffusion rates may be transported largely by active transport. Strategies to bypass crowding are discussed below.

### Strategies for Small Molecules

We define small molecules as any molecule below the molecular weight of 100 kDa (∼5 nm radius), and here, we discuss movement of this size class of proteins. In neurons, MTs form bundles separated from each other by about 25 nm in the axon (by Tau) and by about 65 nm in the dendrite (by MAP2) (Chen et al., 1992; Méphon-Gaspard et al., 2016). Tau cross-links between different MTs are transient, and Tau is known to diffuse along the MT lattice (Hinrichs et al., 2012). Separation of 25 nm between axonal MTs is unlikely to allow entry of large organelles or molecular complexes within the MT bundle. Moreover, this deep axonal region is rich in neurofilaments and actin that can be as many and as closely spaced as MTs (Osborn et al., 1978; Ganguly et al., 2015). However, the diameter of neurofilaments (6–10 nm) is lower than that of MTs (25 nm) (Fuchs and Cleveland, 1998). Thus, the deep axonal space may preferentially be available for protein diffusion both along MTs and in the cytosolic spaces between MTs and other cytoskeletal elements (Figure 3E).

**FIGURE 3:** Strategies to maintain cargo movement that can bypass physical crowding. **(A)** Multiple active motors can increase pulling force or reverse. **(B)** Motors can switch to a MT track that is less crowded. **(C)** Macromolecular complexes can be transported by transient association with organelles interspersed potentially with diffusion. **(D)** Switch to an actin track from a MT track. **(E)** Small soluble proteins can preferentially diffuse deep within the axon (arrows indicate diffusion) rich in MTs and other cytoskeletal elements. Some MAPs can also diffuse along MTs. These proteins can evade crowding near the axonal cortex.

Soluble proteins, such as Casein Kinase 1 (CK1) and Ca^2+^/calmodulin-dependent protein kinase IIa (CamKIIa), are also actively transported. Soluble proteins are actively transported in two ways: by associating with synaptic vesicles as shown for CK1 (Gross et al., 1995) and CamKIIa (Scott et al., 2011), and by associating with molecular motors as shown for choline acetyltransferase that directly binds to Kinesin-II (Sadananda et al., 2012). Due to transient association with MBOs and their small size, soluble proteins undergo assisted movement characterized by bouts of processive transport followed by periods of classic diffusive behaviors (Figure 3C) (Smith and Simmons, 2001; Kuznetsov et al., 2009; Scott et al., 2011). Although intermittent active transport may reduce the overall speed of transport as compared to continuous active transport at large distances (>100 μm), the ability to diffuse buffers soluble proteins from MT-based crowding factors.

Macromolecular crowding can have consequences on proteins that use assisted transport depending on the protein’s turnover rate in the axon. The turnover rate of a protein measures the time when half the existing protein is replaced with newly synthesized protein. This depends on the half-life of the protein, the rate of its synthesis, and rate of its transport. Fast turnover proteins like CK1 (half-life ∼16 h) (Cohen et al., 2013) may be more susceptible to the slowing down of transport from physical crowding along the transport path compared to CamKIIa, which is known to have a longer half-life (∼2 days) (Cohen et al., 2013). This difference in susceptibility may arise from the degradation of fast turnover proteins before it reaches the distal part of the neuronal process. Radioisotope pulse-labeling reveals the presence of proteins such as tubulin and neurofilament proteins for at least 45 days post labeling along the neuronal process (Lasek R., 1968; Lasek R.J., 1968; Brown et al., 1982; Nixon et al., 1982). One possible explanation for long lifetimes of proteins in the axon as found by radioisotope labeling (Lasek R.J., 1968; used in Lasek R., 1968; Brown et al., 1982; Nixon et al., 1982), in contrast to stable isotope labeling with amino acids in cell culture (SILAC) (used in Cohen et al., 2013) based labeling, may be due to the axon having a slower degradation rate compared to the cell body or synapse.

In summary, small molecules may preferentially diffuse deep within the axon, but also associate intermittently with organelles leading to active transport. Depending on the turnover rate of the protein, multiple modes of transport can assist in maintaining the levels of any given protein at the distal end of the neuron.

### Molecular Motor-Based Strategies for Large Molecular Complexes

Large macromolecular complexes may be too large for substantive diffusive transport in axons given cytosolic viscosity. Therefore, the transport of molecular complexes may occur largely by active transport. Some examples of molecular complexes include the ribosomal machinery (25–30 nm) (Schavemaker et al., 2017) and the proteasome machinery (20S proteasome ∼15 nm, 60S proteasome diffusion coefficient ∼0.44 μm^2^/s) (Unno et al., 2002; Ritland Politz et al., 2003). One way to transport large macromolecular complexes is to move the components individually and then assemble them distally. One such example is the ribosome whose components can be assembled in a nucleolus-independent manner in the axons where both the individual ribosomal proteins and their mRNAs are independently actively transported in the axon (Elvira et al., 2006; Noma et al., 2017; Shigeoka et al., 2018).

Another way to transport large macromolecular complexes includes association with an MBO. An example is a pre-assembled proteasome known to associate with MBOs that leads to its processive transport (Otero et al., 2014). The interaction of the pre-assembled proteasome with MBOs is regulated through the adaptor protein PI31 (Liu et al., 2019). Since the size of molecular complexes is of the order of small vesicles, the types of crowding agents affecting these molecular complexes while undergoing active transport are likely to be similar to those faced by MBOs. However, due to a half-life of 4–7 days of the proteasome subunits (Cohen et al., 2013), constant active transport may not be required. Large molecular complexes with slower turnover are likely to be more resilient to local transient crowding.

Unlike large protein complexes, RNAs are transported by aggregating into a Membrane-Less Organelles (MLOs) with the help of RNA binding proteins (RBPs) (Lin et al., 2015; Gopal et al., 2017; Maharana et al., 2018). RNAs have a high negative charge and naked RNA has an extended geometry (Borodavka et al., 2016) both of which are unfavorable for diffusion-dependent movement in the cytosol (Lifland et al., 2011). RNAs such as β-actin >500 kDa in size, ∼1.5 kb in bp length and ∼12 nm in physical length (Borodavka et al., 2016) are known to have very low diffusion coefficients (Lifland et al., 2011). RBPs such as TDP-43, hnRNP A2, FUS (Shan et al., 2003; Fujii et al., 2005; Gopal et al., 2017) can condense RNA and form MLOs. These MLOs are known to be actively transported by MT motors (Kanai et al., 2004; Turner-Bridger et al., 2018). In contrast to protein complexes and organelles, MLOs are highly dynamic and undergo fission and fusion events while interacting with each other (Gopal et al., 2017). These deformations may allow MLOs to transport mRNAs through crowded locations by changing their size and geometry, thus bypassing some physical crowding bottlenecks.

Active transport appears to be the primary means through which large macromolecular protein complexes or RNA-protein complexes move along axons. Thus, the ability of such complexes to navigate crowding are likely similar to those used by MBOs (see below). Additionally, dynamic MLOs that can deform can permit easier movement across crowded regions in the axons.

### Molecular Motor-Based Strategies to Help Organelles Navigate Crowded Locations

In the above-mentioned cases, physical crowding can act as a deterrent to the movement of proteins and larger cargo. Molecular motors are a primary means to help MBOs and MLOs bypass physical crowding (Goychuk et al., 2014; Lakadamyali, 2014). Distinct features of molecular motors allow them to help cargo maneuver across physical obstacles typically along the tracks that they use. These obstacles may be present on the MTs, such as MAPs, or present in the cytosol around the MT such as MLOs and MBOs. The strategy used depends on the types of molecular motors that a specific cargo use.

Motors can be distinguished based on the type of cytoskeletal filament they walk on (MT or F-actin). These motors include kinesins, dyneins (MT dependent) (Vale et al., 1985; Schroer et al., 1989) and myosins (F-actin dependent) (Mehta et al., 1999). Specific properties of motors can help cargo maneuver across crowded regions of the neuron. Mechanisms to overcome crowding on MTs can include: (i) dissociation of kinesin on encountering MAPs or other kinesins on the MT, as shown for Kinesin-1 (Telley et al., 2009); (ii) binding to multiple MT protofilaments/MTs, which may allow the cargo to switch to another less physically crowded protofilament on the same MT or to switch to another MT (Figure 3B) (Hunt and Howard, 1993); (iii) dissociating with an increased frequency from MT plus ends as shown for Kinesin-3, that may prevent traffic jams along the MT (Leduc et al., 2012; Guedes-Dias et al., 2019); (iv) frequent protofilament switching as is shown for dynein, that can help cargo navigate across physical obstacles (Reck-Peterson et al., 2006); and (v) a physically obstructed MT-attached cargo may switch to the F-actin cortical ring via unconventional myosin V that allows cargos to move tangentially to the MT bundle and access a less physically crowded region of the axoplasm (Figures 1A, 3D) (Ali et al., 2008; Vassilopoulos et al., 2019). Thus, a combination of the above-mentioned characteristics of molecular motors can allow transported organelles to circumvent physically crowded locations along MT tracks.

Cargos such as endosomes can recruit multiple motors, such as kinesin and dynein (Figure 3A) (Welte, 2004; Vershinin et al., 2007; Hendricks et al., 2010). Multiple motors are able to exert a greater pulling force (Rai et al., 2013) that may allow organelles to continue moving despite plasma membrane drag or other cytosolic obstacles. Computational modeling suggests that the presence of MTs in close proximity is sufficient to recruit multiple motors on different MTs (Conway et al., 2014; Wortman et al., 2014). Moreover, *in silico* modeling also suggests that a combination of increased pulling force and track switching due to kinesins engaged on multiple MTs is sufficient for sustained cargo transport across organellar traffic jams (Lai et al., 2018). Cargos are also known to recruit opposing motors (Rogers et al., 1997; Ally et al., 2009; Encalada and Goldstein, 2014). This can lead to frequent switching of direction (viz. reversals) of motion (Morris and Hollenbeck, 1993; Welte et al., 1998; Encalada and Goldstein, 2014). Reversing cargos may be able to sample many more MTs owing to dynein’s ability to switch MT protofilaments while walking (Wang et al., 1995; Reck-Peterson et al., 2006; Hoeprich et al., 2017). Increased MT sampling may, in turn, help cargos maneuver across obstacles present on MTs, and potentially in the cytosol as well. Indeed, reversals have been observed in multiple systems for multiple types of cargo (Welte, 2004; Hendricks et al., 2010). These cargo reversals may also distribute the cargo along the track and maintain a steady supply to the distal ends (Wu et al., 1998). The cytoskeletal network physically crowds the neuron and creates space constraints for organelle trafficking while providing the tracks required for movement. Mechanisms such as multiple motors, multiple tracks, and opposing motors are all strategies that use this contiguous cytoskeletal physical crowding in an advantageous manner to circumvent physical crowding on tracks or crowding from other organelles.

The neuronal cytoskeleton consists of regularly spaced (∼200 nm) braid-like actin cortical rings (Figure 1A) (Xu et al., 2013; Vassilopoulos et al., 2019), actin filaments deep in the axoplasm (Ganguly et al., 2015), neurofilaments within the axoplasm (Friede and Samorajski, 1970; Fuchs and Cleveland, 1998), and a staggered array of MTs of lengths from 1 to 10 μm in *C. elegans* and up to 760 μm in *Mus musculus* (Chalfie and Thomson, 1979; Bray and Bunge, 1981; Tsukita and Ishikawa, 1981). The cytoskeletal arrangement may be disrupted by external forces caused, for instance, through body movement that subjects the underlying neuronal processes to tensile and torsional forces. These stresses can induce local deformations in the neuronal process, which may disrupt active transport and result in non-uniform crowding (Ahmed et al., 2012, 2013). Neurons can resist deformations by maintaining the stiffness of the MT bundle through cross-linking between MTs (Peter and Mofrad, 2012). Furthermore, uniform membrane tension allows the axon to regain its shape after deformation, a process thought to depend on axonal spectrin (Krieg et al., 2014, 2017; Dubey et al., 2019). Thus, recovering from deformation of the axon after movement and reducing deformation maintains neuronal shape and potentially helps in maintaining local cargo transport.

## Effects of Physical Crowding in Neurodegeneration

Neurodegenerative diseases due to a combination of genetic predisposition, environmental factors, and traumatic injuries are a confluence of multiple factors such as pathogenic aggregates, defects in transport, and collapse of the axonal cortex (Trapp et al., 1998; van Horssen et al., 2011; Sorbara et al., 2014; Kreiter et al., 2018). Many neurodegenerative diseases are known to be initiated by the formation of macromolecular aggregates (Kumar et al., 2016), mutations in MT motors and their adapters (Morfini et al., 2009a; Millecamps and Julien, 2013; Okamoto et al., 2014), and increased concentration of reactive oxygen species (ROS) (Williamson and Cleveland, 1999; Manoharan et al., 2016). These defects further lead to (i) mitochondrial and lysosomal dysfunction (Bros et al., 2014; Gowrishankar et al., 2015), (ii) changes in the cytoskeleton of the neuron (Dubey et al., 2015; Oberstadt et al., 2018), and (iii) stalled MBO and MLO transport (Baloh et al., 2007; Morfini et al., 2009a; Burk and Pasterkamp, 2019). We discuss below the sub-cellular consequences of some neurological disorders whose pathologies can influence or be influenced in part by physical crowding, and their likely consequences on cargo movement.

### Crowding in Neurodegenerative Diseases

Abnormal aggregate formation of some RBPs (like TDP-43 and FUS) or structural proteins (like Tau and α-Synuclein) are characteristics of neurodegenerative diseases like frontal temporal dementia (FTD) and amyotrophic lateral sclerosis (ALS) for the former two (Neumann et al., 2006; Cairns et al., 2007; Vance et al., 2009; Mackenzie et al., 2010), and familial Alzheimer’s and Parkinson’s diseases for the latter two (Alonso et al., 1996; Polymeropoulos et al., 1997). Increase in the size of aggregates over time is seen with Tau where the formation of 20–40 nm granular aggregates precedes larger 200 nm neurofibrillary tangles (Maeda et al., 2007). Tau oligomers can form granular aggregates up to 200 nm in diameter, or fibrils that are up to 1 μm in length and 20 nm in diameter (Maeda et al., 2007). RBPs generally form dynamic aggregates within cells (Brangwynne et al., 2009; Lin et al., 2015; Maziuk et al., 2017), which are hypothesized to become gel-like when transitioning to form pathological aggregates in neurons (Gopal et al., 2017). These RBP containing aggregates are seen to increase in numbers along the axon in diseased neurons (Fang et al., 2014). Different types of aggregates (amorphous, ribbon-like, fibril, etc.) (Figure 4C) that are formed in the neuron have been thought to lead to divergent disease phenotypes (e.g., ALS, FTLD-TDP-A, and FTLD-TDP-C) (Laferrière et al., 2019) that may arise from altering different cellular processes (e.g., recruitment of proteasome, interaction with MBOs, etc.) (Fahrenkrog and Harel, 2018; Guo et al., 2018). Dysfunctional aggregated Tau has been shown to (i) decrease binding of kinesin to MTs (Stamer et al., 2002; Mandelkow et al., 2003; Cuchillo-Ibanez et al., 2008), (ii) disrupt MT bundles (Figure 4D) (Lovestone et al., 1996; Shemesh et al., 2008), and (iii) crowd the neuronal process (Alonso et al., 1996; Wegmann et al., 2018). Decreased MT bundle stability may also result in the collapse of the space between MTs (Figure 4E) that in turn leads to loss of soluble-protein diffusion within the MT bundle, reducing movement of material to the synapse.

**FIGURE 4:** Defects observed in neurodegenerative diseases. **(A)** Defective transport or increased physical crowding leads to increase in stalled cargo by disengaging motor-based transport as indicated by arrows. **(B)** Increased aggregation of cytosolic proteins lead to increased viscosity in the entire neuron. **(C)** MLOs may undergo a phase transition from a fluid to a gel-like state which further crowds the neuron as illustrated by the arrow. **(D)** Discontinuous coverage of MTs throughout the axon or **(E)** collapsed MT bundle lead to jamming of cargo due to unavailability of tracks and defects in cytosolic protein diffusion respectively in the neuronal process.

Despite independent origins of the above aggregates, all of them have the potential to alter physical crowding in the neuron. Small aggregates of Tau, α-Synuclein, and TDP-43 formed during disease initiation is associated with reduced trafficking of MBOs and MLOs (Ebneth et al., 1998; Lee et al., 2006; Alami et al., 2014). Indeed, overexpression of proteins such as α-Synuclein that form pathogenic aggregates leads to a decrease in transmembrane and cytosolic pre-synaptic proteins at synapses (Kamal et al., 2001; Stamer et al., 2002; Scott et al., 2010). This is consistent with the hypothesis that the presence of aggregates itself may physically impede cargo movement. The presence of protein aggregates may alter neuronal trafficking through both a disruption of specific cellular pathways as well as an increase in physical crowding.

Many animal models for neurodegenerative disease that resemble human late-onset neurodegenerative diseases are associated with an increase in the number of stalled MBOs, MBOs that travel shorter distances before stalling, and a decrease in the number of transported MBOs (Gunawardena and Goldstein, 2001; Stamer et al., 2002; Pigino et al., 2003; White et al., 2015; Kreiter et al., 2018). Transport defects in models of late-onset neurodegeneration may arise from three different processes: (i) a slow buildup of reduced MBO transport (Williamson and Cleveland, 1999; Duncan and Goldstein, 2006), (ii) an increase in intracellular viscosity with age (Figure 4B) (Lamoureux et al., 2010), and (iii) a loss in regulation of the transport machinery (Figure 4A) (Morfini et al., 2009b; Falzone et al., 2010). These altered processes can, independently or synergistically with increased physical crowding, contribute to the progressive nature of the disease with aging. However, all three different processes can also directly increase physical crowding in the neuron and promote further cargo stalling. The sources of age-dependent increase in viscosity are currently unclear. Further investigation is necessary to distinguish between the relative contributions of cargo stalling and viscosity changes in worsening of late-onset neurodegenerative diseases.

Nearly all these diseases progress through an increase in crowding in the neuron. Defects in cargo transport in diseased neurons are thought to starve the distal ends of the neuronal process of freshly synthesized proteins and cargo (Collard et al., 1995; Gunawardena and Goldstein, 2001; Mandelkow et al., 2003; Pigino et al., 2003; Scott et al., 2010; Okamoto et al., 2014). These defects in cargo transport could partly occur through increased physical crowding, which subsequently reduces, over time, the material reaching the synapse. Progression of many neurodegenerative diseases that result in death of a neuron is associated with axonal swellings and “dying-back” of the neuron from its distal end. Dying back may occur due to starvation of the distal neuronal ends of different types of materials transported from the cell body (Schiffer et al., 1994; Collard et al., 1995).

### Crowding in Brain Injury and Demyelination

Axonal swellings are also seen in cases of physical injury [e.g., traumatic brain injury (TBI)] (Rand and Corville, 1934), or where the myelin sheath is inflamed and destroyed (e.g., demyelinating diseases like multiple sclerosis) (Trapp et al., 1998; Ohno et al., 2014). These external factors lead to increased swelling due to disruption in the cytoskeleton (Datar et al., 2019), or damage due to increased local ROS (Trapp et al., 1998; Ohno et al., 2014). TBI exerts large rotational and stretch forces that can lead to axonal buckling and local swelling (Figure 5i.A). These local swellings are hypothesized to occur due to loss of membrane tension through disruption of MT-membrane interactions (Datar et al., 2019). These swellings may act temporarily as locally uncrowded regions, where material can freely diffuse (Figure 5i.B). However, over time these periodic swellings have bent and non-uniform MTs that begin depolymerizing 3 h post-injury (Tang-Schomer et al., 2012). The disruption of MT tracks leads to loss of transport at this local swelling, leading to an accumulation of vesicles and proteins (Shemesh et al., 2008; Hooman et al., 2009; Johnson et al., 2013). This accumulation of MBOs in the swelling can further reduce transport and diffusion rates due to physical crowding of the region (Figure 5i.C). Severe TBI is associated with a higher risk of Alzheimer’s disease later in life (Fleminger et al., 2003; Li et al., 2017). This increased risk may arise from the injury site continuing to act as a locally crowded region that favors aggregation of organelles and aggregation-prone proteins. This potential for increased crowding may be one factor that contributes to the observed increased risk of Alzheimer’s in TBI patients (Figure 5i.D). Demyelination diseases are caused by a loss of myelin (Figure 5ii.A), essential for electrical conduction (Hess and Young, 1952; Yin et al., 2006). Survival of demyelinated neurons has been shown to require redistribution of mitochondria to the demyelinated region to scavenge locally increased ROS (Mahad et al., 2008; Ohno et al., 2014). Mitochondria have been shown to slow down or stall transport of other organelles (Che et al., 2016; Sood et al., 2018). Thus, redistribution of a large organelle like a mitochondrion could physically occupy significant available space in the cross section of a narrow diameter axon (Figure 2), and this crowding may be followed by additional reduction in transport by reducing the available space for other MBOs and MLOs to move through this region (Figure 5ii.B). Mitochondrial redistribution is an early event in disease progression and may initiate physical crowding (Bilsland et al., 2010; Sorbara et al., 2014). Mitochondria appear sufficient to physically crowd the neuron and stall other cargos in the vicinity (Che et al., 2016; Sood et al., 2018). As demyelination progresses, ovoids filled with organelles and altered MT structures are formed (Figure 5ii.C) (Trapp et al., 1998; Ohno et al., 2014). The local varicosities filled with organelles, similar to that seen in TBI, lead to secondary axotomy (Trapp et al., 1998). Therefore, loss in myelin of the neuron can lead to local physical crowding which in turn is one factor among many that may disrupt the trafficking of material from the cell body to the synapses (Figure 5ii.D). The protective movement of mitochondria in the early stages of disease comes along with a potentially detrimental effect of increased physical crowding. In space-constrained axonal processes, this balance is a tradeoff between competing effects. Whether this crowding tradeoff is actively monitored, and if so, how it occurs, is worth investigating.

**FIGURE 5:** Sub-cellular events after injury/disease leading to axonal swellings. **(i.A)** Large tensile or torsional forces can buckle the cytoskeleton of the axon leading to local swelling of the axonal membrane. **(i.B)** Axonal swellings are temporarily locally uncrowded and allow free diffusion of proteins as indicated by lighter green. **(i.C)** Eventual accumulation at the time scale of minutes of organelles and destabilization of MTs in the swelling can lead to a loss of the movement of organelles and proteins illustrated by a darker shade of green. **(i.D)** Axonal swelling further may act as a locally crowded region promoting aggregation of proteins that later in life may predispose the neuron to degeneration. **(ii.A)** In the case of demyelinating diseases, external factors lead to a redistribution of mitochondria along the axons. **(ii.B)** Increase in mitochondria in a region may lead to increased crowding in its vicinity that reduces movement of organelles and cytosolic proteins as illustrated by a darker shade of green. **(ii.C)** Reduced movement of organelles and proteins at a region leads to swelling of the plasma membrane. **(ii.D)** Axonal swelling filled with organelles can lead to increased disruption of transport.

## Perspective

A mounting body of evidence suggests that intracellular physical crowding is an inevitable consequence of the geometry and content of the axon (Pannese et al., 1984; Méphon-Gaspard et al., 2016; Sood et al., 2018; Vassilopoulos et al., 2019). Physical crowding in healthy neurons is not detrimental to neuronal health (Sood et al., 2018), perhaps in part due to molecular motors that have ways to circumvent locally crowded regions while carrying cargo over large distances (Hunt and Howard, 1993; Reck-Peterson et al., 2006; Telley et al., 2009; Guedes-Dias et al., 2019). However, any increase in physical crowding, as seen in multiple neurodegenerative diseases from classical tauopathies to TBI, may underlie some of the pathological changes that are observed in these conditions. Neurons seem to be the most adversely affected by aggregate-prone proteins such as Tau and RBPs (Spillantini et al., 1997; Neumann et al., 2006), even though these proteins are present in many cells (Gu et al., 1996; Hoell et al., 2011; Tollervey et al., 2011). The susceptibility of neurons to physical crowding might arise from the narrow diameter of the axon compared to the diameter of transported organelles, bundled MTs that exclude organelles between them, a continuously varying and dynamic cytoskeleton, stalled organelles, and actin-rich regions (Osborn et al., 1978; Chalfie and Thomson, 1979; Misgeld et al., 2007; Assaf et al., 2008; Encalada and Goldstein, 2014; Krieg et al., 2017). In healthy neurons, local crowding may not have detrimental consequences. However, in unhealthy neurons, increased crowding may explain the observation of reduced cargo movement over time (Williamson and Cleveland, 1999; Stamer et al., 2002; Mandelkow et al., 2003). Further, local crowding amongst other changes may lead to trafficking defects of multiple cargos over time (Evans et al., 2003; Sugiyama et al., 2008). Delineating the contribution of individual crowding agents toward overall physical crowding as impacts cargo movement or protein diffusion may help shed light on neurodegenerative disease progression.

However, crowding is not all detrimental. Neurons show multiple trade-offs in terms of function and crowding. MTs may crowd the neuronal process by excluding organelles from within the MT bundle, but the presence of the bundle provides structural integrity to the neuronal process (Peter and Mofrad, 2012) and enables MT motor-dependent transport (Vale et al., 1985; Schroer et al., 1989). Organelles by their size and geometry cause crowding, but are essential for neuronal function e.g., synaptic vesicles and mitochondria. Large organelles like mitochondria can physically crowd the neuronal process, but their presence at nodes of Ranvier and at synapses are critical for neuronal function (Ly and Verstreken, 2006; Chiu, 2011). Further, Tau aggregates crowd neurons in tauopathies, but may also protect neurons from ROS-mediated damage (Lee et al., 2005). Nonetheless, the density of organelles, and even protective aggregates formed during neurodegenerative diseases, may need to strike a balance. Too much physical crowding over time may adversely affect cargo movement (Hooman et al., 2009; Kuznetsov and Avramenko, 2009) where the ability of molecular motors to circumvent crowding fall short for the degree of physical crowding seen in unhealthy neurons. *In vitro* studies with defined physical crowding due to Tau have identified a precise degree of physical crowding on MT tracks where molecular motors are unable to sustain cargo displacement (Hagiwara et al., 1994; Stern et al., 2017; Shigematsu et al., 2018). Similar studies with other MAPs or crowding agents may help delineate the contribution of crowding to progressive slowing down of organelle transport in neurodegenerative diseases.

Physical crowding can also be utilized by the neuron to promote the distribution of cargo throughout the neuronal process via slowing down of transport using physical barriers. Indeed, cargo such as synaptic vesicles and mitochondria are seen to distribute along the entire neuronal process, often at actin-rich regions (Frederick and Shaw, 2007; Kang et al., 2008; Iacobucci et al., 2014; Sood et al., 2018; Sure et al., 2018). These can lead to formation of naturally occurring cargo reservoirs that can be mobilized during cellular need (Hoerndli et al., 2015; Sood et al., 2018), such as during neuronal injury, where mitochondria localize to the cut-site (Han et al., 2016; Zhou et al., 2016), or during repeated stimulation of the neuron where synaptic vesicles are mobilized to synapses (Kittelmann et al., 2013; Hoerndli et al., 2015). Therefore, physical crowding is an inevitable consequence of the cellular design of axons but may be co-opted to distribute cargo along the neuronal process.

One way to reduce crowding in neurodegenerative models may be to gently perturb the MT and actin cytoskeleton. Cytoskeletal elements such as actin and MT physically crowd the neuronal process while maintaining the shape of the neuron, as well as enabling transport. Low doses of paclitaxel that stabilize MTs (Horwitz, 1994) have been shown to reduce axonal swellings in a hereditary spastic paraplegia model (Fassier et al., 2013). One potential explanation is that drugs that target the MT cytoskeleton may be able to provide additional tracks for transport, thereby alleviating crowding. Further, a low dose of such drugs in combination with treatments to reduce aggregation have been shown to slow disease progression in patients (Trojanowski et al., 2005; Zhang et al., 2005). This slowing of neurodegeneration may in part occur through reduced physical crowding in neurons.

To understand neurodegenerative disease progression, it is valuable to understand the effect of increased molecular crowding on the movement of different proteins and organelles. Currently, most studies have focused on movement of MBOs and MLOs by molecular motors (Cairns et al., 2007; Mackenzie et al., 2010; Encalada and Goldstein, 2014; Fang et al., 2014; Gowrishankar et al., 2015). We speculate that diffusive movement may also be altered, contributing to deprivation of proteins at distal ends of unhealthy neurons. It is interesting to note that diffusion at longer distances is slower than predicted by experimentally observed diffusion of the same proteins at shorter distances (Saxton, 1994; Masuda et al., 2004). Therefore, experimental paradigms that assess diffusion at short length scales have to be used in conjunction with those that can assess diffusion at longer length scales. To investigate the contribution of crowding to diffusive transport of proteins at short length scales, one can use fluorescence correlation spectroscopy (FCS) (Dauty and Verkman, 2004; Banks and Fradin, 2005) and single particle tracking (SPT) (Hall and Hoshino, 2010). FCS and SPT can assess differences in rates of diffusion dependent, for instance, on the density of organelles in the vicinity of the diffusing proteins. Further, studies using magnetic resonance imaging (MRI) have been used to calculate the apparent diffusion coefficient of water *in vivo* (Sener, 2001; Trouard et al., 2008). The diffusion coefficient of water has been suggested to depend on multiple factors, including the caliber of the axon (Assaf et al., 2008). MRI based imaging can help assess diffusion at longer length scales and is particularly suited for *in vivo* studies (Sener, 2001). To assess long-term rates of active transport of MBOs without using radioactive tracers, experiments such as Retention Using Selective Hooks may be useful (Boncompain et al., 2012; Farías et al., 2016; Li et al., 2016). This method is particularly valuable as it might be able to bridge the gap between vesicle imaging over short-time scales of minutes and movement of cargo over hours that result in observed steady state distributions of cargo. Using this method one can begin to assess the role of crowding, for instance, from microtubule-based crowding agents and actin on long-term cargo movement in neurons. The above methods may also allow screening for drugs that aid in alleviating crowding while concomitantly increasing movement of cargo in neurons.

Several studies are necessary to understand the role of physical crowding in the neuron on both diffusive and active transport. Additionally, understanding how crowding changes during neuronal injury or neurodegenerative disease and whether it has both protective and detrimental effects are all open to investigation. Physical crowding effects may be as important as molecular pathways in progression of neurodegenerative diseases.

## Author Contributions

SK conceived the study. VS and SK wrote the manuscript.

## Conflict of Interest

The authors declare that the research was conducted in the absence of any commercial or financial relationships that could be construed as a potential conflict of interest. The reviewer AK declared a past collaboration with one of the authors, SK, to the handling Editor.
